# SS-SWT and SI-CNN: An Atrial Fibrillation Detection Framework for Time-Frequency ECG Signal

**DOI:** 10.1155/2020/7526825

**Published:** 2020-05-18

**Authors:** Hongpo Zhang, Renke He, Honghua Dai, Mingliang Xu, Zongmin Wang

**Affiliations:** ^1^State Key Laboratory of Mathematical Engineering and Advanced Computing, Zhengzhou Science and Technology Institute, Zhengzhou 450003, China; ^2^Cooperative Innovation Center of Internet Healthcare, Zhengzhou University, Zhengzhou 450001, China; ^3^School of Information Engineering, Zhengzhou University, Zhengzhou 450001, China; ^4^Institute of Intelligent Systems, Deakin University, Burwood, VIC 3125, Australia

## Abstract

Atrial fibrillation is the most common arrhythmia and is associated with high morbidity and mortality from stroke, heart failure, myocardial infarction, and cerebral thrombosis. Effective and rapid detection of atrial fibrillation is critical to reducing morbidity and mortality in patients. Screening atrial fibrillation quickly and efficiently remains a challenging task. In this paper, we propose SS-SWT and SI-CNN: an atrial fibrillation detection framework for the time-frequency ECG signal. First, specific-scale stationary wavelet transform (SS-SWT) is used to decompose a 5-s ECG signal into 8 scales. We select specific scales of coefficients as valid time-frequency features and abandon the other coefficients. The selected coefficients are fed to the scale-independent convolutional neural network (SI-CNN) as a two-dimensional (2D) matrix. In SI-CNN, a convolution kernel specifically for the time-frequency characteristics of ECG signals is designed. During the convolution process, the independence between each scale of coefficient is preserved, and the time domain and the frequency domain characteristics of the ECG signal are effectively extracted, and finally the atrial fibrillation signal is quickly and accurately identified. In this study, experiments are performed using the MIT-BIH AFDB data in 5-s data segments. We achieve 99.03% sensitivity, 99.35% specificity, and 99.23% overall accuracy. The SS-SWT and SI-CNN we propose simplify the feature extraction step, effectively extracts the features of ECG, and reduces the feature redundancy that may be caused by wavelet transform. The results shows that the method can effectively detect atrial fibrillation signals and has potential in clinical application.

## 1. Introduction

Atrial fibrillation (AF) is the most common arrhythmia. The estimated number of individuals with atrial fibrillation globally in 2010 was 33.5 million [1]. More than one-third of the patients diagnosed with atrial fibrillation are asymptomatic [2, 3]. In other words, they are usually diagnosed until visiting a hospital. Although atrial fibrillation does not represent a fatal disease itself, the presence of atrial fibrillation increases the risk of strokes and death [4], posing a burden on social public health services [5–8]. Screening for atrial fibrillation in asymptomatic patients has been suggested as an effective method to reduce the risk of this disease; however, the early detection of atrial fibrillation remains problematic. For example, paroxysmal atrial fibrillation usually only lasts for a few heartbeats which makes it time consuming for manually reading ECG waveforms [9]. Therefore, the early detection of patients with asymptomatic atrial fibrillation through the AF screening and preventive anticoagulant therapy is of considerable significance to reduce the risk of cardiovascular events in the case of a stroke [10].

In this paper, we combine the time-frequency features of ECG signals with the convolutional neural network using the specific-scale stationary wavelet transform (SS-SWT) we propose. By designing SI-CNN: an atrial fibrillation detection framework for the time-frequency ECG signal, we effectively achieve the rapid and automatic detection of atrial fibrillation signals. The main contents of this paper are summarized as follows:

- In this paper, we propose a method for extracting time-frequency features of ECG signals for convolutional neural networks, which we call “specific-scale SWT (SS-SWT).” It is different from the time-frequency feature extraction in common deep learning fields. After the ECG signal is decomposed using a stationary wavelet transform (SWT), the approximation coefficients of specific scales are selected as valid information and converted into a 2D time-frequency coefficient matrix for the input of the CNN. The decomposed scales and selected scales are determined according to the characteristics of the ECG signal. As SS-SWT simplifies the step of signal feature extraction, there is no need to perform denoising, debaseline drift, and other operations. At the same time, on the basis of retaining the effective information of the ECG signals, SS-SWT reduces the amount of data and data redundancy.
- In conjunction with SS-SWT, we design the scale-independent convolutional neural network (SI-CNN) specifically for the 2D time-frequency coefficient matrix of ECG signals. Unlike a square or rectangular convolution kernel used in common CNN, a strip convolution kernel with height 1 is used in this paper, which preserves the frequency domain independence between each scale after SS-SWT, fusing the time domain features. Compared with other algorithms in the same field, SI-CNN is more in line with the characteristics of the coefficient matrix generated from the specific-scale stationary wavelet transform (SS-SWT). The proposed method has provided technical support for real-time monitoring of atrial fibrillation.

The rest of this paper is divided into four sections.  Section 2 introduces the research status of AF recognition in related fields. In Section 3, the details of the proposed SS-SWT and SI-CNN in this paper are introduced.  Section 4 introduces the experiment results and then compares the automatic detection framework of atrial fibrillation proposed in this paper with other algorithms. Finally, Section 5 summarizes the full text and looks forward to future work.

## 2. Related Work

Atrial fibrillation is characterized by the rapid and irregular movement of the atria. There are two main manifestations on the electrocardiogram: one is that the P-wave disappears and is replaced by an irregular and high-frequency f-wave (up to 350–600 Hz) [11]; the other is the distance between the R-wave peaks of the adjacent ECG signals (RR interval) changes irregularly [12]. Therefore, the current ECG recognition technology for atrial fibrillation by ECG is mainly divided into the following two categories: analysis based on atrial activity and analysis based on ventricular activity. The method based on P-wave characteristics relies heavily on the accurate detection of P-waves and f-waves. Henriksson et al. proposed a new method for assessing the signal quality index (SQI) for atrial fibrillation detection, which facilitates the analysis of atrial fibrillation signals in noisy ECG signals [13]. Tang et al. developed a hybrid Taguchi-genetic algorithm (HTGA) that facilitates Gaussian decomposition of ECG signals and extracted P-wave morphological features to detect atrial fibrillation [14]. However, the low signal-to-noise ratio characteristic of low-amplitude f-waves makes atrial activity analysis error prone. This problem is alleviated in an analysis based on ventricular activity by the easy-detecting high amplitude of the ECG QRS complex. Therefore, methods based on irregular RR interval features are widely used in atrial fibrillation detection. Lian et al. proposed an atrial fibrillation detection algorithm based on the variation of the RR interval [15]. Zhao et al. measured atrial fibrillation entropy for atrial fibrillation detection in the time window of a short RR time series [16]. Peimankar and Puthusserypady used a random forest classification algorithm based on the RRI, RMSSD, nRMSSD, and other features extracted from the RR interval to achieve an accuracy rate of 97.86% in 300 heartbeats [17]. However, many methods based on ventricular activity require long pieces of data to identify long AF events (20-s) and are limited in dealing with very short AF events [18]. At the same time, the performance of these algorithms highly depends on the detection of P-wave or R-wave peaks. If the relevant peak is detected incorrectly or erroneously, its accuracy may decrease.

In recent years, some atrial fibrillation detection algorithms based on handcrafted features have been proposed. Zhou et al. designed a recursive algorithm for real-time automatic detection of atrial fibrillation based on nonlinear/linear integer filters, symbol dynamics, and Shannon entropy extracted by RR intervals [19]. Asgari et al. used stationary wavelet transform to extract features in ECG signals and support vector machines to detect atrial fibrillation. This method does not require the location of P-wave or R-wave peaks [20]. García et al. introduced a method of detecting atrial fibrillation in ECG signals of various lengths based on relative wavelet energy (RWE) [21]. Though many handcrafted features rely on expert knowledge, they may not represent the best characteristics of the ECG signal. In addition, due to the specificity of the handcrafted features, the accuracy and efficiency of these methods under different datasets may vary greatly, so these methods fail to be used widely clinically.

A deep neural network is an artificial neural network [22], which has been applied to image recognition [23], drug discovery [24], medical image analysis [25], and other fields. In addition, deep learning is widely used in the field of bioinformatics [26]. They produce results that are comparable to human experts and, in some cases, superior to human experts [27]. Deep learning extracts abstract features from ECG signals, frees up the reliance on handcrafted features, and does not require expert knowledge. Andersen et al. combined CNN with LSTM and used the RR interval extracted from 30 heartbeat lengths to achieve an accuracy of 97.80% under the MIT-BIH atrial fibrillation database [28]. Furthermore, deep learning is used in many studies to extract abstract features from ECG signals and to get rid of the dependence on handcrafted features. Yildirim et al. employed the MIT-BIH arrhythmia database segmented into 10-s ECG signals and used a one-dimensional convolutional neural network to classify 17 diseases including atrial fibrillation [29]. Pourbabaee et al. designed a five-layer convolutional neural network to identify five-minute ECG data, achieving good results under the PAF database [30, 31].

In order to better extract the characteristics of ECG signals, many atrial fibrillation detection methods combined time-frequency features with deep learning have been proposed. There are many common time-frequency methods, such as short-time Fourier transform [32], continuous wavelet transform (CWT) [33], modified frequency slice wavelet transform (MFSWT) [34], and stationary wavelet transform (SWT) [32]. These methods convert 1D ECG timing signals into 2D time-frequency features and feed these features to the classifier. Xu et al. proposed an automatic AF beat detection framework, combining a modified frequency slice wavelet transform (MFSWT) and a convolution neural network [34]. He et al. developed a method combining continuous wavelet transform (CWT) and 2D convolutional neural network for atrial fibrillation detection [33].

Using time-frequency features of ECG signals is a very effective way to extract the characteristics of ECG signals. However, there are also some problems in the current research. First, the frequency domain interval of each ECG signal waveform is limited. After the time-frequency transform, some of the frequency band information is redundant. Keeping the redundancy parts increases the complexity of the system, poses a higher calculation burden, and also reduces the robustness of the algorithm. Meanwhile, most of these methods that combine time-frequency characteristics with deep learning use the time-frequency transform to convert ECG signals into images and then identify them with the idea of image recognition. On the one hand, directly converting the signal into a three-channel RGB time-frequency image increases the amount of data, thereby greatly increasing the amount of neural network operations. On the other hand, this combination is simply a splicing of the two methods and does not make good use of the characteristics of both time-frequency features and deep neural networks. Among them, Xia et al. went one step further and directly regarded the coefficient matrix of the ECG signal after stationary wave transform as a gray-scale “image” and sent it to the neural network they proposed [32]. They obtained better results than the direct time-frequency transform from ECG signals to pictures for classification. Inspired by this article, we improve the existing deep learning methods based on time-frequency features and design a deep learning framework for the time-frequency characteristics of AF signals. The framework achieves good results in identifying AF signals in 5-s ECG segments.

## 3. Methods

Figure 1 shows the flowchart of the atrial fibrillation detection framework proposed in this paper. This framework is mainly divided into three parts, namely, signal preprocessing, feature extraction “SS-SWT,” and AF signal classification “SI-CNN.” The preprocessing section cuts the original ECG signals into fixed-length segments and normalize them to prepare for feature extraction. In the second stage of feature extraction, each ECG signal segment is converted into a two-dimensional coefficient matrix using a stationary wavelet transform (SWT), and a specific scale coefficient is selected as valid information to feed into the next stage. The third stage is the classification of the signals. The SI-CNN model proposed in this paper is used to train the data to complete the classification of the AF signals.

### 3.1. Data Preprocessing

The incoming ECG signal is first cut into 5-s segments. In order to improve the effectiveness of feature extraction and the robustness of the network, we normalize each ECG signal after cutting and transform it between −1 and 1. This study focuses mainly on the identification and detection of atrial fibrillation signals. Therefore, the signals are classified into two types: AF signals and non-AF signals. A threshold parameter *P* is used to determine the classification to which each segment of the signal belongs [9]: if the atrial fibrillation signal contained in a segment reached the value of *p* or more, the segment is classified as an atrial fibrillation signal. The *p* value selected in this study is 0.5.

In addition, in the next step of feature extraction, the stationary wavelet transform of the signal requires a specific number of signal sampling points. For instance, a *j*-scale SWT of a signal requires the signal length to be a multiple of 2^*j*^. In this paper, the zero-padding process is performed before the SWT is performed.

### 3.2. Feature Extraction

Feature extraction is crucial in deep learning and is the basis of deep neural networks. A good feature extraction process should minimize the data complexity on the basis of retaining the effective features of the data because a smaller input data can achieve a higher calculation speed. In this paper, we propose an effective feature extraction method for ECG signals, and we call it specific-scale stationary wavelet transform (SS-SWT). It uses the stationary wavelet transform (SWT) to convert a time-series ECG signal into a 2D coefficient matrix, selects the specific scales of parameter, and feeds the matrix into the proposed CNN.

Wavelet transform's good spatial-and-frequency-domain localization characteristics make it possible to analyse the signal in both the time domain and the frequency domain and effectively extract the information in the signal. The basic definition of the wavelet transform is as follows:

(1) WTfa,τ≤ft,ψa,τt≥1a∫fRtψt−τdt,

where *a* is the scale factor and *τ* is the translation factor. Furthermore, *ψ*_*a*,*τ*_(*t*) is the wavelet basis function, as shown below:

(2) $$\begin{array}{c} \psi_{a,\tau }\left(t\right)=a^{-\left(1/2\right)}\psi \left(\frac{t-\tau }{a}\right)a>0,\;\tau \in R. \end{array}$$

Wavelet transform is divided into continuous wavelet transform (CWT), discrete wavelet transform (DWT), and stationary wavelet transform (SWT). When *a* and *τ* are continuous values, it is a continuous wavelet transform (CWT). However, because of the continuity of the continuous wavelet transform scale, the delay is high and there is a considerable amount of redundancy during the calculation. At the same time, most signals are given in a discrete setting (e.g., ECG signals used in this work), a discrete wavelet transform (DWT), or a stationary wavelet transform (SWT) is sufficient for these signals. A discrete wavelet transform (DWT) samples the signal in different resolution when it is decomposed. It produces different length of wavelet coefficients in each scale. A stationary wavelet transform (SWT) does not downsample the signal at each scale, and the time resolution of each scale is the same, retaining most of the valid information of the signal. The wavelet transform decomposition produces a matrix of coefficients, which is very suitable as the input of a CNN. In this study, a stationary wavelet transform is used to process the signal. For the stationary wavelet decomposition, each scale bisects the frequency domain of the signal and produces a detail coefficient (D) and an approximation coefficient (A). At the next scale, the approximation coefficient produced by the previous scale is used, and the decomposition is performed again. The coefficients of each scale include the energy-scale information of the scale corresponding to the frequency-domain window. Since the detail coefficients of each stage are decomposed from the approximation coefficients of the previous stage, after performing a *j*-scale wavelet transform, it is only necessary to reconstruct all the detail coefficients and the approximation coefficients of the last stage to recover all the information of the original signal.

Figure 2 shows the data processing of the SS-SWT we propose. The raw ECG signal shown in Figure 2 is transformed into 1 approximation coefficient and 8 detail coefficients after an eight-scale stationary wavelet decomposition. We choose db5 as our wavelet basis function.

The different scales of coefficients of the ECG signal after SWT represent its different frequency domain characteristics. Moreover, the effective features of ECG signals are mainly included in several specific scales. Therefore, in this paper, we use SS-SWT to extract the features of the signals, in other words, after wavelet decomposition of the signal, only certain scales of coefficients are selected and send to the next neural network. According to the Nyquist sampling theorem, the frequency domain of the ECG signal with a sampling rate of 250 Hz is 0–125 Hz. In this paper, we use the 8-scale stationary wavelet transform to decompose the original ECG signal to obtain 9 groups of wavelet coefficients, which represent the following 9 frequency bands: 62.5–125 Hz, 31.25–62.5 Hz, 15.63–31.25 Hz, 7.81–15.63 Hz, 3.91–7.81 Hz, 1.95–3.91 Hz, 0.98–1.95 Hz, 0.49–0.98 Hz, and 0–0.49 Hz. In these frequency bands, the effective information of the ECG signal is mainly concentrated in 0.5∼40 Hz, and the remaining frequency intervals are mainly interference information such as baseline drift and noise. It can be seen that the coefficients on the D2–D8 scale included the frequency domain interval in which the valid information of the ECG signal is located, so we choose the wavelet coefficients on the seven scales of D2–D8, and the signals on the remaining two scales, D1 and A8, are discarded. The 8-scale wavelet decomposition is chosen because it can effectively isolate these valid information. The low-scale decomposition cannot separate the baseline drift interference (0–0.5 Hz), while the higher-scale decomposition is not necessary. In order to better show the effective information contained in the selected scale, in Figure 3, we show the signal obtained by reconstructing specific scales of the coefficients generated by the ECG signal after SWT, where 3(a) is the original ECG signal, 3(b) is the reconstructed signal generated by D1–D8 coefficients, and it can be seen that the baseline drift of the signal in 3(b) is removed, and 3(c) is the signal reconstructed by the D2–D8 scales of the coefficients. It can be seen that the signal contains valid information in the original signal, and most of the high-frequency noise and baseline drift interference are removed. It can be seen that SS-SWT retains the valid features in the ECG signal and removes the invalid information.

### 3.3. Architecture of the Proposed SI-CNN

After SS-SWT mentioned above, a wavelet coefficient matrix at specific scales containing valid information is passed to the network for learning.  Table 1 gives the structure and parameters of the neural network proposed in this paper in detail. As can be seen from the table, the network designed in this paper consists of 5 groups of similarly structured layers. Each group contains two consecutive convolutional layers, a maximum pooling layer, a batch normalization layer, and a dropout layer. After this 5 sets of layers, we use a global average pooling layer instead of the common fully connected layer. After that it is a fully connected layer and finally a softmax layer to output the results. The batch normalization layer and the dropout layer are used for reducing overfitting, improving gradient propagation, and increasing learning speed, while the global average pooling layer is used instead of the traditional fully connected layer because the global average pooling layer does not require a lot of training and tuning parameters like the fully connected layer, and reducing the spatial parameters will make the model more robust and the anti-overfitting effect is better.

A classical CNN is consisted of alternating superimposed convolutional layers and max-pooling layers. In the convolutional layer, the features and their associated weights were extracted by means of local connections. The weight of each layer of the convolution kernel parameters is trained using a backpropagation error algorithm. The larger the number of convolutional layers, the larger the number of relevant features are extracted. The sigmoid or tanh nonlinear activation function is then applied to the convolution feature. The nonlinear activation function is calculated as follows:

(3) $$\begin{array}{c} y_{i}^{k}=\sigma \left(W^{k}x_{i}+b^{k}\right), \end{array}$$

where *W*^*k*^ and *b*^*k*^ are the weights and the offsets of the *k*^*th*^ convolutional feature map, respectively; *x*_*i*_ is the input to the kth convolutional layer; and *y*_*i*_^*k*^ is the output of the kth convolutional layer. In this study, the ECG signal after the stationary wavelet transform become a coefficient matrix, which can be approximated as a gray-scale “image” and feed in a 2D CNN. However, unlike ordinary images, for the coefficient matrix in this study, the data of each line were the wavelet coefficient of the ECG signal at a certain scale, and the wavelet coefficients of each scale are independent from each other between the rows. Unlike in a normal image, the convolution between rows in the convolutional layer is obviously not in line with the actual situation. Therefore, we use a convolution kernel with a height of 1 to fuse only the data in the row direction. In the convolution, each line still maintained its data independence. The same pooling operation is also performed in the pooling layer. This operation better fused the features after the stationary wavelet transform, conforms to the characteristics of the wavelet transform coefficient matrix, and does not cause aliasing of effective information, and we call it scale-independent CNN (SI-CNN).

In this study, two consecutive convolutional layer stacking methods using 1 × 3 convolution kernels are used in the convolution strategy. Compared to a single-layer convolution kernel, two consecutive 1 × 3 convolution kernels have the same receptive field as a 1 × 5 convolution kernel as shown in Figure 4, and the continuously stacked convolution layer increases the depth of the network. At the same time, the continuous 1 × 3 convolution layers have more nonlinearity than a 1 × 5 convolution, making the decision function more decisive.

## 4. Results and Discussion

### 4.1. Experimental Setup

The SI-CNN model proposed in this paper is run under the Keras platform based on the Tensorflow1.8 framework. The device is a Razer PC running Windows 10. The device has an i7 7700HQ CPU and 16 GB memory. To shorten the training time for deep learning, the device also has an NVIDIA GForce 1060 graphics card and 6 GB video memory. The average time required to train a single period of the model is approximately 50 s. The initial experiments show that the model converged after 35–50 training periods; therefore, 50 periods are used in this study to ensure the complete convergence of the model and limit the chances of overfitting.

### 4.2. Experimental Data

The dataset used in this experiment is from the MIT-BIH AFDB [35, 36]. There are 25 sets of two-lead ECG records in the MIT-BIH AFDB, each with a duration of 10 hours and 15 minutes and a sampling rate of 250 Hz. We use this database to classify the atrial fibrillation signals in this study. The original data of “00735” and “03554” cannot be obtained. In the remaining dataset, there are 605 segments containing four types of ECG segments, of which 291 segments are atrial fibrillation signals, 14 segments are atrial flutter signals, 12 segments are junctional rhythm, and 288 segments are other rhythms.

According to the preprocessing method above, we cut each record in AFDB into 5-s fixed-length segments, and 168667 ECG data are cut out, of which 67243 are atrial fibrillation signals and 101424 are non-AF signals. The non-AF signals include the atrial flutter signals, junctional rhythm, and other rhythms.  Figure 5 shows our division of the training set, validation set, and test set. According to the ratio of 7 : 1 : 2, we divide the training set, validation set, and test set, and the data proportion in each dataset remains the same.

### 4.3. Evaluation Index

For the experiment results of this study and comparison with other experiments, we first calculate true positives (TP), false negatives (FN), true negatives (TN), and false positives (FP). On the basis of these four parameters, the sensitivity (Se), specificity (Sp), and overall accuracy (Acc) are calculated to evaluate the results of this study. These metrics are calculated as follows:

(4) $$\begin{array}{c} \text{Se}=\frac{\text{TP}}{\text{TP}+\text{FN}}\times 100\%,\\ \text{Sp}=\frac{\text{TN}}{\text{TN}+\text{FP}}\times 100\%,\\ \text{Acc}=\frac{\text{TP}+\text{TN}}{\text{TP}+\text{FP}+\text{TN}+\text{FN}}\times 100\%. \end{array}$$

In this study, the adaptive estimation, also known as the Adam optimization algorithm, is used to optimize the model. Adam is different from the traditional stochastic gradient descent (SGD). The stochastic gradient descent uses a single learning rate to update the total weight during the training process. It is crucial to set the appropriate learning rate as it does not change during the entire training process. However, selecting the right learning rate is increasingly difficult. In detail, a very small learning rate leads to slow convergence, while a very high learning speed may hinder convergence and cause the loss function to fluctuate at a minimum. In addition, if the model falls into the saddle point, the gradient of the model in all dimensions will be zero, so SGD may be difficult to escape. The Adam algorithm has considerable advantages over the other types of random optimization algorithms. Therefore, the Adam algorithm was used to optimize the model.

Overfitting is a common problem in machine learning. The deep learning model has a high degree of complexity, which not only fits the relationship between the input signal and the category label, but also fits the random error and signal noise. To prevent overfitting, we introduce dropout layers into the CNN model we propose. The principle of dropout can be simply understood as discarding some neurons with probability *x* while training. To alleviate overfitting, we add dropout layers to the CNN network structure. In order to test the best performance against overfitting, the dropout rate from 0.1 to 0.4 is tested separately. The test result is shown below.  Figure 6 shows the convergence of training and verification when the dropout rate is set to 0.1, 0.2, 0.25, 0.3, and 0.4. It can be seen from the figure that when the dropout is selected to be 0.1, the model shows obvious overfitting, that is, the verification loss has risen significantly after reaching the lowest point. When dropout is set to 0.4, the accuracy of the model is poor. When the dropout is set to 0.2, 0.25, and 0.3, the performance of the model is not much different. However, it can be seen that when the dropout is set to 0.25, both the loss and accuracy achieve good performance, thus we set the dropout in the model for 0.25.

At the same time, we also compare the impact of different batch sizes on network performance, as given in Table 2. In this article, we finally select a batch size of 128 to obtain the best network effect. In addition, the initial learning rate used in this study is 0.001, and *β*_1_ and *β*_2_ of the Adam optimization algorithm are set to 0.9 and 0.999, respectively. The other parameters in the network are given in Table 3.

## 5. Results

Figure 7 shows the convergence performance of the method used in this study.  Figure 7(a) shows the convergence performance of the proposed method.  Figure 7(b) shows the loss performance of the proposed method. It can be seen that although the result of the training set is slightly better than that of the test set, the model has converged and achieves high accuracy in 50 batches. There is no typical overfitting phenomenon; for instance, the performance of the training continues to increase, and the performance of the test set stagnates (or worsens).

In order to better evaluate the performance of the proposed algorithm, we presented a comparison of the proposed algorithm with other algorithms from the same field using AFDB, as given in Table 4. In this study, we select the following five parameters of atrial fibrillation signals: signal length, methodology, sensitivity (Se), specificity (Sp), and overall accuracy (Acc). The table shows a comparison of the results obtained in this study with those reported in other papers from the same field.

The confusion matrix results of this study are shown Figure 8. As shown in Figures 7 and 8, the sensitivity (Se), specificity (Sp), and overall accuracy (Acc) of the atrial fibrillation recognition algorithm based on the specific-scale stationary wavelet transform (SS-SWT) and the scale-independent convolutional neural network (SI-CNN) proposed in this paper reaches 99.03%, 99.35%, and 99.23%, respectively.

Although the methods used by Tateno and Glass [37], Dash et al. [9], Babaeizadeh et al. [38], Huang et al. [39], Ladavich and Ghoraani. [40], and García et al. [21], are different, they all need to detect the R-wave of the ECG signal. The accuracy of these algorithms is highly dependent on the accuracy of the R wave detection algorithm. When the performance of the waveform detection algorithm is not ideal, these methods find it difficult to achieve better performance. In addition, these methods require a longer signal length.

He et al. [33] used a continuous wavelet transform (CWT) to extract the time-frequency feature of the signal, but the method also relied on the detection of the R wave peak. The peak annotations in the AFDB were used directly to obtain the RR interval information. In the work by Xia et al. [32], the method using a stationary wavelet transform (SWT) achieved a higher result. Different from our work, the proposed algorithm performs an elliptical bandpass filter to remove the baseline drift before performing the stationary wavelet transform. All approximation coefficients and detail coefficients are used simultaneously in the convolution process which in our opinion is not necessary.

This paper has made corresponding improvements to the above points and proposed SS-SWT and SI-CNN: an atrial fibrillation detection frame for the time-frequency ECG signal.

During the SS-SWT, the coefficients at specific scales were selected as valid information, so that we do not need a denoise process. At the same time, the SI-CNN specifically for the ECG signal coefficient matrix also better combines the advantages of SWT and CNN.

In summary, the SS-SWT and SI-CNN proposed in this paper are not dependent on waveform detection and they achieve a high accuracy. At the same time, compared with the same type of time-frequency feature extraction algorithm, the SS-SWT and SI-CNN combine the effective features of SWT and CNN and better preserve the original features of ECG signals. Furthermore, the independence among the various scales of the coefficient matrix is more in line with the characteristics of the ECG signal. From the results, the method of this paper has better performance.

## 6. Conclusion

This paper proposes SS-SWT and SI-CNN: an atrial fibrillation detection framework for the time-frequency ECG signal. In order to better match the input of CNN, we use a stationary wavelet transform to convert the 5-s ECG signal into a time-frequency coefficient matrix. Then, we design a convolutional neural network and a convolution kernel structure for the time-frequency characteristics of ECG signals and effectively extract the time-frequency characteristics of ECG signals to achieve fast and accurate detection of AF signals. The validity and efficiency of the proposed method are verified on the MIT-BIH AFDB dataset. Compared with the existing methods, our method has achieves better results with simpler operation steps and deeper network layers. Therefore, the proposed method has a high clinical potential, and it is the focus of our future work.

## Figures and Tables

**Figure 1:** Flowchart of the proposed framework.

**Figure 2:** Flowchart of SS-SWT.

**Figure 3:** Comparison of signals obtained by reconstructing information at different scales of coefficients. (a) Original ECG signal. (b) Reconstructed signal by coefficients of D1–D8. (c) Reconstructed signal by coefficients of D1–D8.

**Figure 4:** Receptive field of continuous conv layers.

**Figure 5:** Partitioning of training, validation, and test datasets in this article.

**Figure 6:** Comparison of signals obtained by reconstructing information at different scales of coefficients. Structural optimization. (a) Train and validation accuracy on different dropout rates. (b) Train and validation loss on different dropout rates.

**Figure 7:** Results obtained in this study. (a) Train and validation accuracy iters. (b) Train and validation loss iters.

**Figure 8:** Confusion matrix in this study.

**Table 1:** The detailed architecture of the proposed SI-CNN.

CNN parameters	Volume
1st convolutional layer kernel size	1 × 3 × 32
2nd convolutional layer kernel size	1 × 3 × 32
1st max-pooling layer kernel size	1 × 3 × 32
1st batch normalization layer	—
1st dropout layer rate	0.25
3rd convolutional layer kernel size	1 × 3 × 32
4th convolutional layer kernel size	1 × 3 × 32
2nd max-pooling layer kernel size	1 × 3 × 32
2nd batch normalization layer	—
2nd dropout layer rate	0.25
5th convolutional layer kernel size	1 × 3 × 64
6th convolutional layer kernel size	1 × 3 × 64
3rd max-pooling layer kernel size	1 × 3 × 64
3rd batch normalization layer	—
3rd dropout layer rate	0.25
7th convolutional layer kernel size	1 × 3 × 64
8th convolutional layer kernel size	1 × 3 × 64
4th max-pooling layer kernel size	1 × 3 × 64
4th batch normalization layer	—
4th dropout layer rate	0.25
9th convolutional layer kernel size	1 × 3 × 128
10th convolutional layer kernel size	1 × 3 × 128
5th max-pooling layer kernel size	1 × 3 × 128
5th batch normalization layer	—
5th dropout layer rate	0.25
Global average pooling layer	—
6th dropout layer rate	0.25
The number of neurons in the fully connected layer	128
7th dropout layer rate	0.25
The number of neurons in the softmax layer	2

**Table 2:** SI-CNN training results under different batch sizes.

Batch size	Se (%)	Sp (%)	Acc (%)
64	98.76	99.40	99.15
**128**	**99.03**	**99.35**	**99.23**
256	99.38	99.57	99.08
512	98.92	99.00	98.97
1024	97.99	99.54	98.92

**Table 3:** Optimal CNN parameter set for AF detection.

The CNN optimization parameter	Value
Batch size	128
Epochs	50
Optimizer	Adam
*β*_1_	0.9
*β*_2_	0.99
Initial learning rate	0.001
Dropout	0.25

**Table 4:** Comparison of the performances of AF classification algorithms.

Algorithm	Signal lengths	Methodology	Se (%)	Sp (%)	Acc (%)
Tateno and Glass [37]	50 s	RR interval irregular	94.4	97.2	—
Dash et al. [9]	128 beats	RR interval irregular	94.4	95.1	—
Babaeizadeh et al. [38]	>60 s	RR interval irregular	92	95.5	—
Huang et al. [39]	101 beats	RR interval irregular	96.1	98.1	—
Asgari et al. [20]	9.8 s	SWT + SVM	97	97.1	97.1
Ladavich and Ghoraani [40]	7 beats	P-wave absence (PWA)	98.09	91.66	93.12
García et al. [21]	7 beats	SWT	91.21	94.63	93.32
He et al. [33]	5 beats	SWT	99.41	98.91	99.23
Xia et al. [32]	5 s	SFWT	98.34	98.24	98.29
Xia et al. [32]	5 s	SWT	98.6	97.17	97.74
Proposed framework	5 s	SWT	99.03	99.35	99.23

## Data Availability

The data used to support the findings of this study are included within the article. Further data can be requested from the corresponding author.
